This article has been retracted.

# *In silico* 3D structure analysis accelerates the solution of a real viral structure and antibodies docking mechanism

**DOI:** 10.3389/fmicb.2012.00387

**Published:** 2012-11-06

**Authors:** Motohiro Miki, Kazuhiko Katayama

**Affiliations:** ^1^Department of Virology II, National Institute of Infectious DiseasesTokyo, Japan; ^2^Denka-Seiken Co., LtdNiigata, Japan

**Keywords:** Norwalk virus, monoclonal antibody, x-ray crystallography, *in silico* modeling, cryo-electron microscopy

## Abstract

Norwalk virus (NoV) is responsible for most outbreaks of non-bacterial gastroenteritis. NoV is genetically diverse and show antigenically variable. Recently, we produced a monoclonal antibody called 5B-18 that reacts broadly with NoV genogroup II (GII). We suspected the 5B-18 binds to a conformational epitope on 3D structure of virion. X-ray crystallography showed us that 5B-18 binds to NoV at the P domain, which protrudes from the capsid surface of the virion. However, there seems to be no space that would allow the IgG to approach the virion. To solve this problem, we used cryo-electron microscopy to examine NoV GII virus-like particles (VLPs). The P domain rises up higher in NoV GII than in NoV GI, and it seems to form an outer layer around the virion. Finally, using *in silico* modeling we found the 5B-18 Fab arms and NoV P region are quite flexible, so that 5B-18 can bind the NoV virion from bottom of P domain. This study demonstrates the shortcomings of studying biological phenomenon by only one technique. Each method has limitations. Multiple methods and modeling *in silico* are the keys to solving structural problems.

## THE BASICS OF NORWALK VIRUS

Norwalk virus (NoV) is responsible for most of the outbreaks of non-bacterial gastroenteritis in developed countries and, it is thought, in developing countries as well. Yet, although NoV was identified more than 30 years ago, we know little about their pathogenicity and basic virology (Guix et al., 2007). Studies of NoV have been hampered by the lack of a cell-culture system or a small animal model in which the virus will grow, except murine norovirus that is classified as NoV genogroup V (Wobus et al., 2006).

NoV belongs to the family Caliciviridae. The genus *Norovirus* has only one species, *Norwalk viruses, *with five genogroups (GI–GV). Genogroup GI and II cause most human infections, and they are further subdivided into numerous genotypes (GI.1–8 and GII.1–17; Zheng et al., 2006). The NoV genome is a 7.3 to 7.7-kb positive-sense, polyadenylated, single-stranded RNA molecule. It contains three open reading frames (ORFs): ORF1 encodes a non-structural polyprotein, and ORF2 and ORF3 encode the major and minor capsid proteins, VP1 and VP2, respectively (Jiang et al., 1992; Lambden et al., 1993).

Without an *in vitro* system for propagating the virus, the antigenicity of NoV has been inferred from studies of virus-like particles (VLPs). Nucleic acid-free VLPs self-assemble when the capsid protein is expressed in a baculovirus expression system (**Figure 1A**). The VLPs are assumed to have a similar morphology and, thus, antigenicity as that of the native virions (Jiang et al., 1992). Cryo-electron microscopy (cryo-EM) and x-ray crystal structures of the prototype norovirus VLP (GI.1, Norwalk virus) showed that the VLPs form a T = 3 icosahedral structure (Prasad et al., 1994, 1999).

**FIGURE 1:** **The cryo-EM image of GII.10 VLP and the P dimer structure fit to the cryo-EM image by *in silico* modeling**. The cryo-EM structure of NoV GII.10 VLP was constructed with 180 molecules of VP1 protein **(A)**. The cross-section of GII.10 VLP **(B)**. P domains (blue and green) rise up from shell domain (yellow), and it seemed to construct an outer layer of the capsid. Diagram based on the x-ray crystal structure of the GII.10 P domain-Fab complex shows Fab bound to the lower side of the P1 sub domain. Top side indicates the outside of the VLP, and the shell side contains the VLP core that is called shell. A white arrow indicates the GII.10 P dimer; the monomer is colored blue and purple. Black arrow shows MoAb 5B-18 Fab region. Green represents the heavy chain, and yellow represents the kappa chain. The part of oval shadow represents VLP shell **(C)**. The x-ray crystallography was fit into the cryo-EM structure by *in silico* modeling **(D)**. The GII.10 P domain (apo P domain structure) into the A/B dimer subunit (light blue and pink, respectively) and C/C dimer subunit (cyan).

However, structures of large protein complexes are difficult to determine by x-ray analysis. We sought to understand the structure of the virion and how it interacts with antibodies by combining data from x-ray diffraction, cryo-EM, and *in silico* modeling.

## A MONOCLONAL ANTIBODY REACTS BROADLY WITH NoV GII

NoV is generally detected by RT-PCR with degenerate primers or an ELISA with NoV-specific antibodies. Many polyclonal and monoclonal antibodies used in the ELISA kits were developed in mice or rabbit immunized with norovirus VLPs (Hansman et al., 2011).

Recently, we produced a monoclonal antibody called 5B-18 that reacts broadly with NoV GII (Hansman et al., 2012). In fact, 5B-18 is used as a NoV GII broad-range capture antibody in a commercial ELISA kit [NV-AD(III) SEIKEN NoV antigen ELISA] and in an immunochromatography (IC) kit (Quick naviNoro IC kit, both from Denka-Seiken, Japan).

The 5B-18 monoclonal antibody was produced by immunizing a mouse with norovirus VLPs. Several monoclonal antibodies bind to the shell (S) domain (Yoda et al., 2003; Li et al., 2010), and others bind to the protruding (P) domain (Lindesmith et al., 2012). We suspect that 5B-18 also binds to S or P domain on the surface of the NoV virion. However, no high-resolution structural details of the antibody binding to the VLPs, S domain or P domain are available.

## X-RAY CRYSTALLOGRAPHY OF THE BINDING SITE

The 5B-18 binds major NoV genotypes, such as GII.4 and GII.3, and the minor NoV genotypes GII.10 and GII.12 strongly. We suspect 5B-18 binds to a conserved epitope on the NoV capsid surface. We wanted to define the recognition site of 5B-18 and the NoV minor genotype GII.10 P domain, and we began with x-ray crystallography, one of the gold standard for protein structural studies. We expressed the NoV GII.10 P domain in the *Escherichia coli *strain BL21 (DE3). The P domain was purified and stored in gel filtration buffer. Next we prepared of 5B-18 Fab fragment by immunizing a mouse with NoV GII.4-strain 445 VLPs (GenBank accession number DQ093064; Denka-Seiken, Japan). To prepare crystals of the bound complex, purified GII.10 P domain and Fab were mixed in a 1.4:1 ratio. Crystals were grown by the hanging-drop vapor-diffusion method, mixing the protein and reservoir solution (40% [vol/vol] polyethylene glycol [PEG] 400, 5% [wt/vol] PEG 3350, and 0.1 M acetic acid, pH 5.5) in a 1:1 ratio. Crystals grew over 1 week at 20°C.

One GII.10 P domain-Fab complex crystal diffracted x-rays to a resolution 3.3Å, and we solved the structure by molecular replacement with a GII.10 P domain monomer (PDB ID 3ONU) and a mouse Fab (PDB ID 1WEJ) as search models. Molecular replacement indicated an asymmetrical unit contained two P domain monomers and two 5B-18 Fabs, each with a kappa and a heavy chain (**Figure 1C**; Hansman et al., 2012).

The binding of the P domain and the Fab involved nine hydrogen bonds. Of these, eight linked the P1 subdomain to the kappa chain, and one linked the P1 subdomain and the heavy chain. More specifically, the amino acids in the P1 subdomain amino acids that interacted with the 5B-18 Fab were as follows (in each pair, the amino acids are for the P1 domain and Fab, respectively): Tyr533 and Tyr92 (one bond), Thr534 and Gly93 (three bonds), Thr534 and Trp97 (one bond), Leu535 and Tyr32 (one bond), Glu496 and Tyr92 (one bond), and Asn530 and Ser94 (one bond). Finally, Val433 and Asn52 in the heavy chain formed one hydrogen bond (Hansman et al., 2012).

## CONFIRMATION OF 5B-18 BINDING

With the x-ray crystallographic analysis, we found the 5B-18 antibody bound to a hidden site on the P domain that is located inside of the shell of NoV particle. However, in a previous study, the NoV GI structure indicated that bottom of the P domain was completely covered by the shell of NoV particle (**Figure 1C**). If the structure of GII is the same as GI, then 5B-18 could not bind GII. These results presented an apparent paradox for the 5B-18 binding mechanism. To resolve the paradox, we set out to identify the binding residue in the capsid.

From the crystallographic analysis, we knew that the 5B-18 Fab formed hydrogen bonds with residues at three sites in the P1 subdomain, called A, B, and C (**Figure 2A**). By aligning the amino acid sequences of representatives from NoV GII genotypes, we discovered that Val433 (site A) was the most variable. Other genotypes had threonine, serine, asparagine, leucine, or methionine at this position. Thr534 (site C) was mostly conserved: the only other amino acid at this position was a serine. Glu496 (site B), Asn530 (site C), Tyr533 (site C), and Leu535 (site C) were all highly conserved among the representative GII genotypes.

**FIGURE 2:** **Schematic diagram of NoV VP1 protein and the amino acid alignment of NoV GII VP1 sequences**. Capsid (VP1) sequences from 11 GII genotypes were aligned, and the GII.10 capsid sequence was used as the consensus. The GII.10 P domain residues that interacted with the 5B-18 Fab involved three sites on the P domain termed A, B, and C. The six GII.10 P domain residues that interacted with the 5B-18 Fab are indicated by light blue rectangles **(A)**. Left panel of **(B)**: a schematic of the VP1 deletion mutants. The construct 1 includes the N-terminal region and shell domain of VP1, and amino acids 4–223 from the N-terminal methionine of VP1. The P1-1 and P2 domain constructs without binding site A are construct 2 (amino acids 224–426), with binding site A is construct 4 (amino acids 224–439). Construct 3 has all binding sites A, B and C (amino acids 427–548). Construct 5 deletes binding site A from construct 3 (amino acids 440–548). Right panel of **(B)**: western blotting results with 5B-18. Samples indicated as VLP, NC (negative control), mutant construct 1 (#1), #2, #3, #4 and #5. The black arrow represents VLP band at 58 kDa, and the white arrows represent #3 and #5 products at 13 kDa.

To confirm that 5B-18 binds the A, B, and C regions, we divided the GII.10 capsid domain into three major subdomains: N, S, P1-1 P2, and P1-2. We prepared five constructs (1–5), expressed them in an *E. coli* expression system, and identified a liner epitope of 5B-18 by western blotting (**Figure 2B**). Construct 3, a P1-2 region (i.e., A, B, and C), showed the strongest band signal, and construct 5 (i.e., B and C) showed a positive band. The intensity of the band from construct 5 was only about half the strength of construct 3 because it did not contain epitope A. However, construct 4 included only A, and constructs 1 and 2 also were not detected. Thus, the three 5B-18 epitopes A, B, and C were confirmed to be part of the binding epitope.

Next, we determined if 5B-18 binds to other NoV GII VLPs (**Figure 2A**). We prepared and purified six kinds of GII VLPs that were 809 (GII.3), 104 (GII.4), 445 (GII.6), 026 (GII.10), Hiro (GII.12), and GII.13 VLPs as aligned in **Figure 2A**. The GII VLPs that had all 5B-18 epitopes A, B, and C were captured by the anti-GII VLPs rabbit serum that was pre-coated on ELISA plate and detected with 5B-18 and horseradish peroxidase (HRP)-labeled anti-mouse IgG secondary antibodies. When the cut-off value was under 0.2, 5B-18 detected all kinds of GII VLPs in a dose-dependent manner (data not shown). These results suggested that 5B-18 binds to a variety of GII VLPs. In fact, the commercial ELISA and IC kits use 5B-18 (Denka-Seiken, Japan), and we have practical results showing that 5B-18 detects various infectious NoV GII in stool samples.

## COMBINING CRYO-EM AND *IN SILICO* MODELING TO SOLVE A PARADOX

We had a simple question. Are the structures of NoV GI VLP and GII VLP the same or not? For G1 VLP, there is no space where the 5B-18 can access and bind the bottom of P domain. If the GII VLP had same conformation as the GI VLP, the lower part of the P domain would be buried under the virion shell (**Figure 1C**). However, 5B-18 binds and detects GII VLPs and GII infectious viruses. These conflicting facts suggested that the structures of the GII VLPs and infectious GII virions were different than the GI VLP structure. However, structure determinations by x-ray crystallography have many challenges and limitations, and we suspected this might be one of those cases.

To answer the question, we turned to cryo-EM and *in silico* modeling. We reconstructed the overall structure of GII.10 VLPs and 5B-18 Fabs from the x-ray structural data. To determine if the GII VLP had enough space to allow binding, we also used *in silico* modeling to fit the P and 5B-18 Fabs structures that had been derived by x-ray crystallography.

The GII.10 VLPs formed homogeneous, monodisperse particles in ice. By reference-free class averages and at 10Å resolution (0.5 FSC criterion), these icosahedral particles had several notable features, including spike-like structures extending from the vertices (**Figure 1B**), and at the three- and fivefold axes, significant amounts of the surface of the S domain were exposed (**Figure 1A**). The GII.10 VLP P domain formed a second outer shell that seems to be separated from the S domain by about 15Å (**Figure 1B**). Thus, unlike the GI VLPs and virions, GII VLPs and virions seem to have a space between the shell and bottom of P domain, indicating that the two genotypes have different structures. Furthermore, the electron density was much weaker at the tip of the P domain (the P2 subdomain) than at the base. This observation is consistent with published reconstructions of calicivirus particles (Bhella et al., 2008; Bhella and Goodfellow, 2011) and indicates that the P domains have considerable heterogeneity.

Next we attempted to fit the GII.10 P domain and P domain-Fab complex structures into the GII.10 VLP cryo-EM structure. At 10Å resolution, the GII.10 P domain monomers in the VLP were easily distinguished. We manually fitted the crystal structures of the GII.10 P domain and P domain-Fab complex into the GII.10 VLP cryo-EM map, using published reports of GV.1 P domain dimers and the GV.1 cryo-EM map (Taube et al., 2010) as guides.

We refined the approximate alignment with the Fit-in-Map function in UCSF Chimera (Pettersen et al., 2004) to a cross-correlation coefficient of 0.94 (**Figure 1D**) with excellent results. The x-ray structure of the GII.10 P domain dimer (PDB ID 3ONU) unambiguously fitted the corresponding density in the cryo-EM map (**Figure 1D**). Only some loops of the P2 subdomain did not fit. They had only weak electron density, and their tips were less ordered than the S domain and P1 domains in the cryo-EM reconstruction. These subdomains are probably more flexible. P1, but not the P2, subdomains in the VLP appeared to be connected to the P domain dimers.

Next we fitted the x-ray structure of the P domain from the P domain-Fab complex into the reconstructed A/B dimer subunit and found that the 5B-18 binding site was close to an adjacent dimer of P domain (**Figure 1C**). At the twofold axes, the 5B-18 Fab was hindered by the S domain, which also provided an obstacle to assembly of the neighbor P domain dimer. However, when the P domain was fitted into the C/C dimer subunit, the 5B-18 Fab was in contact with the P domain dimer and slightly interfered with part of the S domain at the fivefold axes. Thus, the antibody binding site overlapped with part of the P1 subdomain.

Thus, this model predicted an unstable structure in which the VLP could not bind with the 5B-18 antibodies. How could this be? There are several possibilities. First, 5B-18 might bind at sites on the P domain that are only transiently exposed. Second, 5B-18 might bind to defects in the P domain. Finally, the Fab arms of 5B-18 might be very flexible.

IgG flexibility is not unknown. For example, a neutralizing antibody 9C12 binds to hexon, the major coat protein of adenovirus, at a ratio of 240 antibody molecules to one virus particle or one antibody per hexon trimer (Varghese et al., 2004). By dynamic light scattering and negative-stain EM, electron-dense material coats the virus, but it was not aggregated at neutralizing ratios. In images reconstructed from cryo-EM, the viral surface was covered by electron density from the 9C12 antibody. Two Fab arms bridge two peripentonal hexons. One has a normal Fab shape and fitted the models well (Harris et al., 1998). The other arm has a somewhat distorted structure. A low-density tail extends to a third hexon that forms a minor alternate binding site. The normal arm binds to a unique site in the asymmetric unit of the virus. It has no alternate binding sites because a penton, rather than a hexon, is positioned at the icosahedral fivefold axis. In addition, the angle between the long axes of the Fabs was <115° that was found in the uncomplexed IgG1 (Harris et al., 1998). Thus, flexibility is important for the bivalent binding of 9C12.

## ESTIMATING THE FLEXIBILITY IN THE STRUCTURE

The findings from the 9C12 study were informative for our 5B-18 paradox. 5B-18 could reach the bottom of the P domain if the Fab domain could bend and escape the P1 subdomain or star-like structure on the shell. 5B-18 IgG bound equally well with intact and partially broken GII.10 VLPs. To determine if 5B-18 binds to intact or broken particles, we took advantage of a characteristic of norovirus VLPs: they are less stable and appear to be broken at high pHs (Ausar et al., 2006). Therefore, we looked at 5B-18 binding at different pHs. At low and neutral pHs (5.3, 6.3, and 7.3), the GII.10 VLPs were mostly homogenous in size and unbroken, but at higher pHs (8.3 and 9.3), they were less homogenous and partially broken. 5B-18 IgG bound to GII.10 VLPs at different pH values with nearly identical efficacies, regardless of the fraction of damaged particles. At pH 5.3, 6.3, and 8.3, the titer was 512,000. At pH 9.3, it was 1,024,000, and at pH 7.3, it was 2,048,000 (optical density cutoff of 0.2; Hansman et al., 2006). We also determined size distribution of the VLPs by dynamic light scattering in each pH conditions. VLPs were shown single peak on diameter 38 to 50 nm (data not shown). These results suggest that 5B-18 appears detects nominally intact GII.10 VLPs.

We studied the 5B-18 binding mechanism by x-ray crystallography, molecular virology, and cryo-EM. We combined the results in *in silico* modeling that simulates molecular dynamics and is a reliable method for revealing fluctuations in protein structure. Each technique complemented the other by filling in for data that was lacking from the others. Interestingly, the 5B-18 study suggests that VLP and viral virion have structure flexibility and that IgG molecule have flexible arms. They co-work each other and bind. *In silico* modeling is clearly a powerful tool for enhancing our understanding of basic viral processes.

## Conflict of Interest Statement

The authors declare that the research was conducted in the absence of any commercial or financial relationships that could be construed as a potential conflict of interest.
